The article "Dietary Restriction and Nutrient Balance in Aging" was published in 2015. Journal: Oxid Med Cell Longev.

# Dietary Restriction and Nutrient Balance in Aging

**DOI:** 10.1155/2016/4010357

**Published:** 2015-11-23

**Authors:** Júlia Santos, Fernanda Leitão-Correia, Maria João Sousa, Cecília Leão

**Affiliations:** ^1^Life and Health Sciences Research Institute (ICVS), School of Health Sciences, University of Minho, 4710-057 Braga, Portugal; ^2^ICVS/3B's-PT Government Associate Laboratory, Braga/Guimarães, Portugal; ^3^Molecular and Environmental Biology Centre (CBMA), Department of Biology, University of Minho, 4710-057 Braga, Portugal

## Abstract

Dietary regimens that favour reduced calorie intake delay aging and age-associated diseases. New evidences revealed that nutritional balance of dietary components without food restriction increases lifespan. Particular nutrients as several nitrogen sources, proteins, amino acid, and ammonium are implicated in life and healthspan regulation in different model organisms from yeast to mammals. Aging and dietary restriction interact through partially overlapping mechanisms in the activation of the conserved nutrient-signalling pathways, mainly the insulin/insulin-like growth factor (IIS) and the Target Of Rapamycin (TOR). The specific nutrients of dietary regimens, their balance, and how they interact with different genes and pathways are currently being uncovered. Taking into account that dietary regimes can largely influence overall human health and changes in risk factors such as cholesterol level and blood pressure, these new findings are of great importance to fully comprehend the interplay between diet and humans health.

## 1. Introduction

The primary molecular mechanisms underlying aging have attracted increased attention, as healthy aging becomes one of the main concerns of the modern society. Cellular activities such as the regulation of metabolism, growth, and aging are modulated by a network of nutrient and energy sensing signalling pathways that are highly conserved among organisms, from yeasts to mammals (reviewed in [1]). Three major signalling pathways involved in longevity regulation have been described: the insulin/insulin-like growth factor (IIS), the Target Of Rapamycin TOR/Sch9 (ortholog of the mammalian S6 kinase), and adenylate cyclase/protein kinase A (AC/PKA). Reducing activity of these pathways is known to promote health and lifespan extension [1]. Signalling through IIS/TOR pathways starts with the binding of ligands, such as insulin and insulin-like growth factor (IGF-1 and IGF-2) in the case of mammals, to specific receptors, which in turn activate the PI3K/Akt/mTOR intracellular signalling cascade that regulates metabolism and stress resistance and consequently aging [2]. Akt kinase directly inhibits the antiaging forkhead FoxO family transcription factor (FOXO), known to regulate autophagy, DNA repair, ubiquitin-proteasome system, and other stress resistance genes [3]. Besides being activated by insulin and IGF-1 via Akt, highly conserved TOR can also respond to dietary amino acids while signalling through other pathways such as the energy sensing pathway AMP-activated protein kinase (AMPK) and sirtuin pathway (SIRT1), downregulating rapamycin-sensitive TOR complex 1 (TORC1) activity. AMPK and SIRT1 are known to mediate longevity in several model organisms in response to dietary regimens [4]. Detailed description of these nutrient signalizing pathways in different models can be found in recently published reviews [5–9].

The study of aging regulating mechanisms can be accomplished by genetic manipulations of these well conserved nutrient-signalling pathways or by using dietary restriction (DR) protocols, in which the intake of one or more macronutrients is reduced without causing malnutrition. One of the best documented DR protocols involves reduction of caloric intake without lack of essential nutrients, termed calorie restriction (CR). The benefits of CR were first described in 1935, by showing that reduced food intake extended lifespan of rats [10]. Since then many studies have demonstrated the beneficial effects of CR on lifespan extension of multiple organisms (yeast, flies, worms, fish, rodents, and rhesus monkeys), as well as on the improvement of overall health in rodent models. However, new evidences have recently emerged from studies in yeast [11, 12] and in higher eukaryotes [13–15] showing the importance of nutrient balance in dietary regimens and its effects on longevity regulation, challenging the notion that the indiscriminate reduction of caloric intake* per se* extends lifespan. These studies increasingly suggest that not only caloric restriction but rather a balance of different nutrients and their ratios have a pivotal role in regulating lifespan [13, 14, 16–18].

In the following sections we start with an overview of different eukaryotic model organisms that allowed establishing the role of metabolic and growth pathways in longevity. The subsequent sections highlight the impact of nutrient balance on the beneficial effects of dietary restriction regimes on longevity regulation and age-related pathologies.

## 2. Aging and Dietary Regimens in Different Eukaryotic Model Organisms

Studies in different eukaryotic model organisms revealed that the pathways regulating metabolism and growth, once active, are also able to modulate aging and increase mortality.

The yeast* Saccharomyces cerevisiae* has been a highly exploited eukaryotic model to study the mechanisms involved in longevity regulation through the assessment of cell survival in stationary phase cultures (known as chronological lifespan—CLS) [19–23]. These studies carried under different nutrient dietary regimens show that reducing glucose concentration in the media (usually from 2% to 0.5 or 0.05%) increase CLS [20, 23–28]. Furthermore, several other single nutrients from the culture medium were also shown to affect longevity regulation (reviewed in [29]). As in higher eukaryotes, in* S. cerevisiae* these nutrients, depending on their abundance, can activate multiple proaging signalling pathways, such as the TOR1-Sch9, primarily activated by amino acids, and the Ras/PKA which mainly responds to glucose but is also regulated by other major nutrients [30–32]. These pathways promote cell division and growth in response to nutrients while inhibiting the general stress response and autophagy [26, 33]. CR further promotes CLS extension in TOR and Sch9p deficient mutants, indicating the presence of other mechanisms in CR-mediated lifespan extension [26]. The Ras/PKA pathway is the primary mediator of the glucose transcriptional response [34] and deletion of* RAS2* causes lifespan extension and stress resistance [35], while imposing CR to long-lived* cdc25-10* mutants (deficient in guanine nucleotide exchange factor that regulates Ras2p activation) does not further extend lifespan of these mutants [36]. Both pathways converge on the stress resistance kinase Rim15p and its downstream transcription factors Msn2p/4p and Gis1p, all of which play key roles in mediating CR effects on longevity [26, 37]. Decreasing TOR-Sch9 signalling also extends CLS in Rim15p independent manner through the modulation of mitochondrial functions. Actually, it has been shown that, in active stages of growth, genetic or pharmacological TOR inhibition results in enhanced mitochondrial coupling, increasing mitochondrial membrane potential and reactive oxygen species (ROS) production that provides an adaptive mitochondrial signal to extend CLS in stationary phase [38, 39]. Others have also reported that CR extends CLS by reducing superoxide anion levels, independently of Rim15p, promoting a more frequent growth arrest in G_0_/G_1_ phase [40, 41]. It has also been shown that mitochondrial respiratory thresholds regulate yeast CLS and its extension by CR, a critical minimum respiratory capacity being crucial for such CLS extension [42].

The role of IIS in aging modulation was first discovered in the nematode* Caenorhabditis elegans* by demonstrating that the phosphatidylinositol 3-kinase (PI3K) signalling cascade is responsible for longevity regulation [43]. Since then, the IIS pathway has been implicated in other biological functions of* C. elegans* [44]. Inhibition of this pathway by using function mutations in* DAF-2*, the only* C. elegans* gene coding for an insulin/IGF-1 receptor ortholog, reduces the aging process [45] and leads to transcription changes of stress response and energy metabolism genes via DAF-16 (FOXO ortholog) [1, 45, 46]. As in yeast, downregulation of the TOR-S6K signalling pathway in* C. elegans* affects longevity by activating stress transcription factors, PHA-4, SKN-1, and DAF-16, which control genes involved in lipid metabolism and autophagy [47, 48]. Also in this model, the IIS and the TOR pathways act in synergy through partially overlapping mechanisms to control longevity [48, 49]. In* C. elegans* the most common dietary restriction protocol to reduce the intake of nutrients, without causing malnutrition (DR), is through the decrease of the bacterial food source, mainly* Escherichia coli*, either by using bacterial dilution, which can extend lifespan from 60% up to 150% [50], or by reducing feeding capability. Increased lifespan is observed in mutants affected in feeding capabilities such as deletion of* EAT-2* (pharyngeal pumping defect) as well as decreased activity of NAC-2 and NAC-3 (gut sodium dicarboxylate transporter) [16, 51, 52]. The study of the role of specific constituents of diet in longevity are still lacking due to the absence of purified diets in* C. elegans*. However, it is known that high glucose diets shorten lifespan in this model by downregulating proteins such as AMPK, FOXO, and glyoxalase [53, 54]. Recently, a glucose transporter that links nutrient restriction and signalling to aging, in this simple organism, has also been discovered. The FGT-1 glucose transporter, a mammalian GLUT-like protein paralog, seems to be responsible not only for transport activity but also for glucose signalling metabolism as reducing its activity increases lifespan to the same level obtained by decreasing DAF-2 signalling [53, 55].

In the fruit fly* Drosophila melanogaster*, reducing IIS signalling by mutations in the insulin-like peptides (DILPS) or insulin-like receptor (INR) shows increased lifespan extension, establishing the role of this pathway as being evolutionary conserved [56]. Direct inhibition of TOR pathway in flies presents a 30% increase in lifespan [57, 58]. However, mutants in the insulin receptor substrate CHICO still respond to DR as do null dFOXO mutants, suggesting only partially overlapping mechanisms for IIS and DR mediated lifespan extension, indicating the existence of other nutrient responding pathways [59, 60]. The usual DR protocol in flies is an* ad libitum* diluted diet, in which the sugar and yeast content can be changed to achieve maximal longevity. In fact, using fixed concentrations of sugar but reducing calories from yeast (protein source) can significantly extend longevity while restriction of dietary sugar yields only modest extension, indicating that protein restriction is more important in lifespan extension in fruit flies [60–62].

As for the other models described above, in mammals, the modulation of the conserved nutrient activated pathways IIS and mTOR, genetically, pharmacologically, or nutritionally, impacts aging and delays age-related diseases. Genetic interventions that limit signalling through IIS pathway in rodents, such as Ames and Snell dwarfs and growth hormone (GH) receptor knockout, are capable of extending lifespan in 50% by diminishing IGF-1 and insulin levels and simultaneously enhance healthspan (reviewed in [5]). Recently, the beneficial effects of CR and IGF-1 levels in longevity are proposed to act through PI3K/Akt/mTOR signalling to reduce mTOR activity, significantly increasing lifespan [2]. The most common DR protocol in mammals is the decrease of calorie intake (CR) which is the most robust dietary intervention to extend lifespan and healthspan in mammals to date. Other DR protocols include protein restriction and intermittent fasting, which do not require a reduction in calorie intake. CR animals have their caloric diet reduced normally 20 to 40% from the* ad libitum* diet given to the control animal and present extended lifespan up to 40% partially by reducing the occurrence of chronic diseases such as cancer, diabetes, and cardiovascular diseases. GH stimulates IGF-1 production, which can be arrested by CR, suggesting that CR uses longevity pathways to limit cancer probably due to energy restriction that alters cell cycle regulation and consequently inhibits cell proliferation and increases apoptosis [63]. CR has also been reported to reduce oxidative damage to DNA, by enhancing the efficiency of DNA repair mechanisms [16, 63]. A schematic illustration of the nutrient-signalling pathways involved in longevity regulation in the different model organisms is provided in Figure 1.

## 3. Nitrogen Sources as Key Effectors on Dietary Regimens

The results in yeast [11, 64] and in higher eukaryotes, described above, clearly favour an emerging perspective where nutrient balance plays a predominant role in the beneficial effects of dietary restriction regimens impacting longevity regulation. Therefore recently several studies tried to clarify which nutrients are affecting longevity regulation and whether they interact. Protein and amino acids have been studied as activators of specific nutrient signalling pathways involved in longevity regulation in multiple model organisms. In the yeast* S. cerevisiae,* dietary amino acid composition has been implicated in CLS regulation. Several studies in the literature report different effects of amino acids on lifespan regulation, dependent on the TOR pathway [19, 21–23, 65]. In this context, it is known that starvation for nonessential amino acids used as preferred nitrogen sources can extend CLS [24, 36, 66], while starvation for essential amino acids reduces CLS [21, 65]. Single amino acids are known to affect longevity and, recently, it has been shown that leucine influences autophagy and extension of CLS during CR [67]. On the other hand, methionine restriction has been described to extend CLS in an autophagy-dependent manner [68] and to confer resistance to multiple cellular stresses through stress-responsive retrograde signalling [69]. Isoleucine, threonine, and valine extend CLS via the general amino acid control (GAAC) pathway [19]. The sensing of certain amino acids, such as leucine, occurs via TOR kinase while the absence of individual amino acids is recognized via GCN2 (general amino acid control nonderepressible 2) [70, 71]. Regulation of these two kinases has been highly implicated in longevity modulation by dietary restriction [72]. Besides amino acids, another nitrogen source commonly used by* S. cerevisiae* such as ammonium (NH_4_^+^) was identified as new key player in the modulation of yeast longevity [73, 74]. These studies reported that NH_4_^+^ is toxic acting as an extrinsic factor affecting yeast CLS, preferentially in amino acid restriction conditions [73]. In extreme CR conditions in water, NH_4_^+^ effects during yeast aging depend on the specific essential amino acid deprived from the medium, with leucine or histidine deprivation being mediated by Tor1p activation and lysine deprivation by Ras2p activation. Sch9p, contrary to Tor1p and Ras2p, mediates cell survival in response to NH_4_^+^ associated with Sch9p-dependent Hog1p phosphorylation [74]. These results suggest that the presence of NH_4_^+^ in the medium (commonly present as the nitrogen source) may be at least partly responsible for the reported decrease in CLS in leucine-starved cells [19, 67]. This work provided new insights into the modulation of CLS by several nutrients, linking NH_4_^+^ toxicity to amino acid limitation [74].

In* C. elegans*, amino acids and proteins are influencing its lifespan through DR. In this scope, it has been shown in a recent study that GCN2, the evolutionarily conserved kinase that directly responds to amino acid deficiency, plays a central role in mediating lifespan extension under DR conditions by converging with TOR/S6K signalling on the PHA-4/FoxA transcription factors and its downstream target genes under stressful conditions [75, 76]. Reducing the uptake of peptides, by Pep-2 deletion, also increases lifespan by reducing insulin signalling [77] and, additionally, mutations in Metr-1/methionine synthase or the use of the common antidiabetic drug metformin, which alters methionine metabolism, is also known to extend lifespan in* C. elegans* [78]. The roles of specific components of the diet in longevity regulation* versus* reduced calorie intake in* C. elegans* are still difficult to elucidate due to the deficiency of purified diets and lack of studies connecting each nutrient contribution and the various pathways implicated in aging.

In* Drosophila melanogaster,* a recent study demonstrated that adding back essential amino acids to DR flies increased fecundity and decreased lifespan back to the full feeding level, while adding back other yeast nutrients, as fatty acids, vitamins, or carbohydrates, add no effect on lifespan nor on fecundity [13]. These results demonstrate that the amount of calories* per se* does not affect lifespan. However, supplementing with methionine by itself increased fecundity to the fully fed level, without reducing lifespan, demonstrating that the assumed tight link between lifespan and fecundity could be uncoupled. Other studies support that methionine and casein supplementation led to extended longevity. On the contrary, a recent study reported positive effects of methionine restriction on longevity in a defined diet, only in the presence of relatively low total amino acids, by downregulating TOR signalling [79]. In order to clarify these different responses to amino acids and in particular to methionine which suggests a possible cross talk between the response pathways of the various amino acids, the use of a fully defined diet such as the complete chemically defined (holidic) diet available for* D. melanogaster* developed by Piper and coworkers [80] has been recommended. The use of this diet has confirmed the positive effects of amino acid dietary restriction on lifespan regulation as well as the negative effect of complete lack of methionine on lifespan extension [61, 80]. This holidic diet is now a promising tool to study the role of individual nutrients in longevity regulation in flies.

As referred above, besides CR, other DR protocols are used successfully in mammal studies on longevity. Recent reports demonstrate that rodents on low protein regimens with 5–15% protein live longer than the ones on high-protein diets with 50% protein intake [14]. This extended longevity due to the fact that protein restriction is associated with reduced mTOR activation, reduced DNA and protein oxidative damage, and reduced spontaneous tumor formation and has been demonstrated to improve renal function [81]. Restriction of single amino acids like methionine and tryptophan has also been described to have a role in longevity regulation in mammals. Studies show that rodents given 80% reduced methionine diet displayed an increase in median and maximum lifespan of 40% in comparison to the controlled fed animals. Methionine restricted rodents exhibit reduced levels of insulin, IGF-1, serum glucose, and mitochondrial ROS, similar to CR restricted animals, although by partially independent pathways [82, 83]. Also, tryptophan restriction has been described to extend mice lifespan by 23% [16] accompanied with delayed sexual maturation and tumor onset and improved hair growth and coat condition. Leucine restriction also appears to be implicated in longevity extension probably by increasing insulin sensitivity via GCN2/mTOR and AMPK pathways [81]. Accordingly, the amino acid sensing pathways GCN2 and mTOR and their cross talk can most probably be implicated in longevity regulation in protein restriction regimens [84].

## 4. Dietary Restriction versus Dietary Balance

As described above, traditional DR differs even within experiments using the same model organism. DR can be implemented by using a diet of constant composition or diets in which the composition varies, either by providing limited food intake or by using a diluted diet. Due to these major discrepancies in DR protocols amongst the major aging models, recent studies have been using the Geometric Framework (GF) approach, consisting of a multidimensional representation of nutrition, in order to better understand the effects of dietary nutrients on feeding behaviour, metabolic health, reproduction, and longevity, among other traits [85]. From these studies emerged the concept that macronutrient ratios between protein and carbohydrates (P : C ratio), but not fat, have key roles in longevity regulation in these models [13, 14, 18, 62]. In fruit flies increased longevity was achieved by reducing the caloric input from the protein source yeast extract. This DR-regimen ameliorated lifespan extension in comparison to isocaloric reduction of sucrose [62]. Similarly, addition of essential amino acids to dietary restriction in sucrose plus yeast-based diet diminishes longevity extension [13]. Another study demonstrated that 1P : 16C diet ratio maximized* D. melanogaster* lifespan, while reduced caloric intake did not extend lifespan [18]. In rodents, increasing the P : C ratio affects longevity without being influenced by total calorie intake, ultimately leading to an increased mTOR activation. The longest lifespan extension was achieved by a low protein high carbohydrate diet, which the authors believe to result from low mTOR activation and low insulin levels. Inhibition of mTOR, a proaging pathway, by manipulating the ratio of macronutrients is believed to extend longevity in rodents [14]. As described above, mTOR and IGF-1 signalling by amino acids and the effect of low protein diets on longevity regulation suggest further investigation into how dietary balance affects aging.

Also in primates, DR composition has a major impact in results regarding lifespan extension, supporting the notion that balance of nutrients in the diet might be more important in healthy lifespan extension than dietary restriction. Two studies, one from the Wisconsin National Primate Research Centre (WNPRC) and another from the National Institute on Aging (NIA) presented different results when subjecting rhesus monkeys to 30% CR regimen. The WNPRC study reported a decreased mortality in the CR group in comparison to the control group with a 50% lower incidence of diabetes, cancer, and cardiovascular diseases [17, 86]. On the other hand, the NIA study did not find significant differences between CR and control groups, although supporting the beneficial impact of CR on healthspan [87]. The major differences between these two studies were the dietary regimens and the protein and carbohydrate sources used in each study. In the WNPRC study, the protein source used was lactalbumin and the carbohydrate source derived from corn, starch, and 28.5% sucrose, whereas, in the NIA study, the protein source used derived from wheat, corn, soybean, fish, and alfalfa meal, and the carbohydrate source derived from ground wheat and corn with 3.9% sucrose [81]. The differences in results from the two studies could be attributed to the variations in food ingredients and possibly to the protein source; one derived from animal and the other derived from plant sources that have been previously described to affect aging [81, 88].

In humans, very recent cohort studies suggest a correlation between age-related diseases and high protein diets from animal sources. Based on the US national survey of health and nutrition, NHANES III database, a recent article reports that the 50-to-65 age group with high protein intake had a 75% increase in overall mortality and a fourfold increased risk of cancer mortality in comparison to individuals with low protein intake, which was attenuated or abolished when protein intake was derived from plants. Interestingly, in individuals over 65 years, the high protein intake was reported to reduce cancer and overall mortality. These results were confirmed in mice, proving that protein absorption is affected by aging. The study also confirms the correlation between higher IGF-1 levels with more dietary protein and the incidence and progression of both melanoma and breast cancer [15]. Likewise, a Swedish cohort reported that low carbohydrate high protein diets are associated with increased risk of cardiovascular diseases [89].

Although the yeast aging model has been pioneer in uncovering many age-related processes, only recently studies addressing dietary balance started to emerge. A recent study shows a nutritional balance occurring between glucose, amino acids, and yeast nitrogen base (YNB) as having a major role in yeast CLS through Sch9p [11]. The same authors have also shown that the ratio between essential and nonessential amino acids greatly affects CLS regulation, in a glucose dependent manner, as a significantly shorter CLS was observed under CR conditions. Methionine restriction and glutamic acid addition were also reported to maximize CLS, and a positive correlation between the additive effects of methionine restriction and glutamic acid addition with CR in CLS was also reported [90]. These reports suggest that also in yeast the well-known CR effect in longevity is strongly dependent on other nutrients in the medium compared to glucose alone. Also, a recent study uncovered how glucose and amino acids (threonine, valine, and serine) modulate stress and aging in yeast [64]. In this study it was reported that, in the presence of glucose, threonine and valine activated TORC1 pathway and serine activated the sphingolipid dependent Pkh1/2 pathway. Both activated pathways converged to active Sch9p which plays a critical role in this nutrient response mechanism. Sch9p seems to be directly involved in nutritional balance in yeast as a new study reports antagonistic effects of* SCH9* deletion on yeast cells grown in synthetic complete medium and natural grape juice, where the nitrogen : carbon ratio significantly differs [91]. In line with these latest results, the CLS shortening under amino acid restriction can be completely reverted by removing nonlimiting good nitrogen sources (NH_4_^+^ or glutamine) from the medium and furthermore NH_4_^+^ is a necessary nutrient for the beneficial effects of CR on longevity to occur [12]. The presence of ammonium is responsible for inducing replicative stress and blocking the consumption of essential amino acids. Furthermore, the negative effects of NH_4_^+^ are mediated by Tor1p, Ras2p, and Sch9p. These results further establish NH_4_^+^ as a key factor involved in the nutritional balance required between nitrogen sources and glucose, to achieve longevity promotion in yeast [12]. A schematic illustration of dietary balance in yeast is provided in Figure 2. These new reports demonstrating that extended lifespan as well as healthspan does not depend only on calorie or dietary restriction but rather on an optimal nutritional equilibrium may have significant acceptance from the general population and a broader application than dietary restriction in worldwide diet regimens [13, 14, 16–18].

## 5. The Interplay between Diet and Age-Related Pathologies

Dietary restriction, as mentioned above, is a potent intervention that increases lifespan and contributes to a lower incidence of chronic diseases, namely, cancer [17, 63]. However, although DR presents high advantages to the aging process and associated diseases, long-term food restriction is unfeasible for most people, therefore presenting low clinical value [92]. Also, inadequate nutrition is known to reduce reproductive function and increase the risk of osteoporotic bone fractures and cardiac arrhythmias [3]. To overcome this low compliance to food DR, a promising strategy is to use DR mimetics, by the development of pharmaceutical compounds that lead to the same physiological effects as DR without significantly reducing food intake. The best studied DR mimetics are rapamycin, metformin, and resveratrol, which have shown anticancer properties and consequently are being tested in clinical trials [63]. Several studies report the effects of metformin, a well-known antidiabetic drug, on reducing spontaneous tumor growth and also increasing the efficacy of radiation in cancer treatment [93, 94]. These beneficial effects of metformin are primarily mediated by the activation of AMPK pathway, known to regulate cellular energy homeostasis, but also by signaling suppression of mTORC1 [63, 93]. The TORC1 inhibitor rapamycin or its analogs induces cell death in breast and colorectal cancer subjected to therapeutic drugs, leading to tumor regression [63]. Resveratrol has been used as CR mimetic known to activate SIRT1 and AMPK with beneficial effects on longevity, cancer, and obesity [95]. The new field of DR mimetics brings to light the vast applications in cancer metabolism and these novel results associating DR mimetics to chemotherapy agents can help reduce the side effects of treated cells by protecting normal cells from stress induced death [63].

Fasting is a dietary regimen that has proven to trigger similar biological pathways as caloric restriction and has gained popularity over the years with people finding it easier to follow than traditional DR. Intermittent fasting (IF) involves restriction of energy intake for periods of 1-2 days a week with no restriction during feeding periods whereas periodic fasting (PF) involves fasting for 3 or more days every 2 or more weeks, also with no restriction during feeding periods. Fasting for a period of 2 or 5 days is known to promote a 50% reduction in glucose and IGF-1 levels in both mice and humans, respectively, and to promote depletion of hepatic glycogen, leading to the generation of ketone bodies [96]. In cancer treatment, fasting has shown to have more consistent positive effects than DR. Fasting generates an extreme environment that induces protective changes in normal cells, but not in cancer cells, that fail to respond to the protective signals of fasting due to the role of oncogenes as negative regulators of stress resistance. This effect is called differential stress resistance (DRS) [97]. On the contrary, long-term DR requires a period of weeks or even months to have some effect and is not capable of achieving high decreases in glucose and IGF-1 levels, besides promoting chronic weight loss, considered detrimental to patients undergoing chemotherapy [63, 96, 97]. Studies in mice have reported that combining fasting cycles and chemotherapy increased cancer-free survival in 20–60% [98, 99] and is effective in improving chemotherapeutic index [100]. Although there are no human data so far, the effect of fasting on enhancing cancer treatment is being tested in clinical trials in both Europe and the USA [96]. IF has also shown major health benefits in both rodents and humans, being able to lower the risk factors associated with metabolic syndrome (MS), such as abdominal fat, blood pressure, inflammation, and insulin resistance, and consequently diminish the risk factor for diabetes and cardiovascular diseases [101–104]. IF can reduce inflammation in rheumatoid arthritis patients and asthma-related symptoms in overweight subjects, inducing significant decreased levels in oxidative stress and inflammation markers [105, 106]. Studies linking IF and cognitive brain function in humans are still scarce; however, recently, dietary patterns have been linked to brain biomarkers of Alzheimer's disease [107]. In fact, in rodent models of Alzheimer's, Parkinson's, and Huntington's disease, IF reduced clinical symptoms, protecting neurons against dysfunction and degeneration by inducing the expression of brain-derived neurotrophic factor (BDNF) [108–110], which suggest that IF interventions could also present benefits in the prevention of brain dysfunction in humans.

Summing up, evidence reported herewith shows that multiple dietary regimens can largely influence overall health and longevity. Nutrient modulating mechanisms are presently being uncovered in different organisms from yeast to mammals, exposing the balance between several nutrients as primordial to aging. These new findings are of great importance to fully comprehend the interplay between diet and humans health.

## Figures and Tables

**Figure 1:** Scheme of longevity regulatory pathways in various model organisms (yeast, worms, flies, and mammals). Identical symbols are used for the orthologous genes in each model organism. In worms, flies, and mammals, dietary restriction reduces signalling through IIS/TOR pathways, deactivating the PI3K/Akt/TOR intracellular signalling cascade and consequently activating the antiaging FOXO family transcription factor(s), known to regulate stress resistance and aging. In yeast, dietary restriction reduces the activity of the TOR/Sch9 and RAS/PKA nutrient-signalling pathways, both converging on the protein kinase Rim15 that in consequence activates its downstream transcription factors Gis1 and Msn2/4, involved in the postdiauxic shift (PDS) element-driven gene expression and stress-responsive elements (STRE) gene expression, respectively. The involvement of RAS signalling in longevity regulation is indicated in the two models where it has been described. lysine (Lys.), methionine (Met.), threonine (Thr.), and valine (Val.). The detailed description and other abbreviations are given in the text.

**Figure 2:** Schematic of nutrients (glucose, amino acids, and ammonium) that accelerate aging through different signalling pathways. A dietary balance between these nutrients is necessary for achieving maximum longevity in yeast. The detailed description and abbreviations are given in the text.
